The article "Naringin Regulates Microglia BV-2 Activation and Inflammation via the JAK/STAT3 Pathway" was published in 2022. Journal: Evid Based Complement Alternat Med.

# Naringin Regulates Microglia BV-2 Activation and Inflammation via the JAK/STAT3 Pathway

**DOI:** 10.1155/2022/3492058

**Published:** 2022-05-19

**Authors:** Li Li, Ru Liu, Jing He, Jing Li, Juan Guo, Yun Chen, Ke Ji

**Affiliations:** ^1^Department of Psychiatry, Hubei Provincial Hospital of Traditional Chinese Medicine, Wuhan 430061, China; ^2^Department of Psychiatry, Hubei Institute of Traditional Chinese Medicine, Wuhan 430074, China; ^3^The Affiliated Hospital of Hubei University of Chinese Medicine, Wuhan 430061, China; ^4^Clinical College of Traditional Chinese Medicine, Hubei University of Chinese Medicine, Wuhan 430074, China

## Abstract

**Objective:**

Microglial BV-2 cells are activated in the brain following insomnia. Naringin (NAR) is a polymethoxylated flavonoid that is also commonly found in citrus fruits and is known for its antioxidant potential. However, the effect of NAR on microglial cells has rarely been studied in the brain of an organism after insomnia. This study aimed to investigate the effects and potential mechanisms of action of NAR on microglial cell activation and inflammation.

**Methods:**

BV-2 cells were obtained from the China Center for Type Culture Collection and randomly divided into five treatment groups: control, model, NAR (10 *μ*M), WP1066 (5 *μ*M), and NAR + WP1066. With the exception of the control group, all groups were stimulated with LPS (1 *μ*g/mL) for 6 h. CCK8 was used to quantify cell viability and a scratch test was performed to detect cell migration. The expression levels of interleukin 6 (IL-6), tumor necrosis factor-alpha (TNF-*α*), interleukin 1 beta (IL-1*β*), nterleukin 10 (IL-10), and insulin like growth factor (1IGF-1) were measured by ELISA. Western blotting was performed to determine the levels of p-STAT3 and p-JAK. The Focalcheck™ Thin-Ring Fluorescent Microspheres kit was used to detect cell phagocytosis. Immunofluorescence was used to observe the expression of iNOS and arginase1 in BV-2 cells.

**Results:**

Compared with the control group, cell migration, cell viability, and the expression of IL-1*β*, IL-6, TNF-*α*, and iNOS were significantly increased in the model group, whereas the expression levels of IL-10, IGF-1, and arginase 1, as well as cell phagocytosis were reduced. With the increase in NAR concentration, cell migration, cell viability, the expression levels of IL-1*β*, IL-6, TNF-*α*, and iNOS decreased, while the expression of IL-10, IGF-1, and arginase 1 increased. Compared with the control group, p-STAT3, and p-JAK expression in the model group were significantly increased (*P*<0.05). Compared with the model group, the expression of p-STAT3 and p-JAK in the NAR, NAR + WP1066, and WP1066 groups was significantly decreased (*P* < 0.05).

**Conclusion:**

NAR treatment inhibited the proliferation, migration, and inflammation of BV-2 cells as well as the activation of microglia to the M1 phenotype. Conversely, NAR treatment promoted the activation of microglia to the M2 phenotype and enhanced the phagocytic function of BV-2 cells by regulating the activity of the JAK/STAT3 pathway.

## 1. Introduction

Insomnia is defined as a subjective experience by patients who are not satisfied with the time and/or quality of sleep and its effect on daytime social functioning. This condition is currently the second most prevalent psychiatric disorder worldwide and may increase the risk of cardiovascular, endocrine, and psychiatric disorders, among others. At present, the pathogenesis of insomnia remains unclear and treatment efficacy is unsatisfactory. Therefore, an in-depth study of the pathogenesis of insomnia is required to improve the efficacy of clinical treatments and the quality of life of patients. Clinical studies have found that lack of sleep can lead to an increase in the number of monocytes, systemic regulation of inflammatory factors, and aggravation of immune dysfunction [1–4]. Lack of sleep can also activate spontaneous innate immunity and STAT family proteins [5]. The mechanism by which immune mediators produced during sleep deprivation destroy the blood-brain barrier, regulate nerve activity, and contribute to nerve damage is poorly understood.

Microglia and astrocytes are the main immune cells of the central nervous system (CNS) and are among the main inflammatory mediators under pathological conditions. Microglia, the innate mononuclear phagocytes of the CNS, are macrophages derived from the embryonic yolk sac that reside permanently in the brain along with neurons, astrocytes, and oligodendrocytes and are referred to as the “macrophages” that colonize the CNS, comprising approximately 10% of the total cells in the adult CNS and function as both immune and phagocytic cells [6]. A number of basic and clinical experimental studies have demonstrated glial activation in the brains of organisms with sleep disorders, including insomnia. Under the stimulation of central nervous system injury or an inflammatory microenvironment, microglia have two types of activated phenotypes M1 and M2. The M1 type produces cytotoxic effects through the production of a large number of inflammatory factors and eventually leads to irreversible loss of neurons. Type M2 promotes anti-inflammation, clearance of dead cells, tissue repair, and reconstruction of extracellular matrix [7]. Pharmacological intervention can significantly inhibit glial activation and the subsequent production of inflammatory factors, thereby alleviating brain nerve injury and ameliorating cognitive impairment triggered by nerve injury [8–12]. Insufficient sleep may cause microglial activation, which promotes an imbalance between proinflammatory and anti-inflammatory molecules and destroys the blood-brain barrier and neurons in the brain tissue [7, 13].

The JAK/STAT3 signaling pathway has been reported to be activated in patients with sleep deprivation and can be regulated in microglia by cytokines, such as IL-6, in the microenvironment. Thus, the JAK/STAT3 pathway is directly involved in regulating the activity of glial and neuronal cells [14–18].

Naringin (NAR) is one of the major active compounds in the herbal formula, Wendan decoction. Okuyama et al. found that NAR could inhibit the activation of microglia and astrocytes, reduce the expression of inflammatory factors in brain tissue, and exert neuroprotective effects [19–21]; however, the underlying mechanism is largely unknown. Therefore, in this study, NAR treatment was assessed at the cellular level, and the effects and mechanisms of action of NAR were studied using pathological, biochemical, and molecular detection methods. Our aim was to provide a theoretical basis for the immunomodulatory and anti-inflammatory activities of NAR in insomnia.

## 2. Materials and Methods

### 2.1. Cell Culture

BV-2 cells were obtained from the China Center for Type Culture Collection (1101MOU-PUMC000063; Wuhan, China). The cells were cultured in RPMI 1640 medium (SH30022.01B; Hyclone; Utah, USA) supplemented with 10% fetal bovine serum (FBS, 10270-106; Gibco) in an atmosphere of 5% CO_2_ and 95% air at 37°C. The medium was replaced every 24 h, and the cells were subcultured or cryopreserved when the confluence reached 70%–80%.

### 2.2. Construction of LPS-Induced Neuroinflammation Model

We constructed a neuroinflammation model based on previous studies [22]. BV-2 cells were divided into five groups: control, model, NAR, NAR + WP1066, and WP1066 groups. The control group was left untreated. The model group was treated with 1 *µ*g/mL of LPS (L118716, Aladdin) and treated for 6 h. The model group cells were divided into three fractions. One part was left untreated, and the other two parts were the NAR group and the NAR + WP1066 group. Subsets of BV-2 cells were treated with NAR (N107344, Aladdin) and/or the JAK2 inhibitor WP1066 (5 *μ*M, S2796, Selleck) [23] for 24 h.

### 2.3. Cell Viability Assay

Approximately 3 × 10^3^ cells were seeded onto in a 96-well plate in RPMI 1640 medium containing 10% FBS and treated with NAR and/or WP1066 for 24 h. To evaluate cell proliferation, 10 *μ*L of Cell counting kit-8 (CCK-8, CA1210, Solarbio) solution was added to each well and the cells were cultured at 37°C for 4 h. Optical density (OD) was measured using a microplate reader (Multiskan FC, Thermo, USA) at 450 nm.

### 2.4. Enzyme-Linked Immuno Sorbent Assay (ELISA)

The expression levels of IL-6 (MU30044, Bioswamp), TNF-*α* (MU30030, Bioswamp), IL-1*β* (MU30369, Bioswamp), IL-10 (MU30055, Bioswamp), and IGF-1 (MU30001, Bioswamp) were measured using an ELISA (Bioswamp; Wuhan, China). Briefly, we diluted the standard, added the sample and enzyme to the test tube, and incubated at 37°C for 10 min after which the reaction was stopped and the OD was measured at 450 nm.

### 2.5. Scratch Test Assay

Cells were seeded onto 6-well plates at a density of 1 × 10^6^ cells/well. Before seeding, four lines were drawn at the bottom of each well 0.5 cm apart using a marker. The following day, a scratch was made perpendicular to the well using a pipette tip against a ruler. The cells were washed with PBS and culture medium was added to the wells. Photographs were taken at 0 and 24 h postscratch to observe scratch healing.

### 2.6. Immunofluorescence

Cells were washed with PBS and fixed with 4% paraformaldehyde for 30 min, followed by treatment with 0.5% Triton X-100 for 20 min at 4°C. Next, the cells were blocked in 5% BSA and incubated with primary antibodies against iNOS (1 : 200, PAB43765, Bioswamp) or arginase 1 (1 : 200, PAB33035, Bioswamp) at 4°C overnight. The next day, the cells were incubated with Alexa Fluor 488-conjugated AffiniPure goat antirabbit antibody (1 : 200, SAB43742, Bioswamp) for 1 h at 37°C and the nuclei were stained with 4′,6-diamidino-2-phenylindole for 10 min at 37°C. Immunofluorescence was observed under a fluorescence microscope (DMIL LED; Leica).

### 2.7. Cell Phagocytosis Assay

Following the addition of 1 *μ*m fluorescent microspheres at cells: microspheres ratio of 1 : 100, 1 × 10^6^ cells were incubated at 37°C with 5% CO_2_ for 30 min. The cells were then washed with PBS and processed according to the manufacturers' instructions for Focalcheck™ Thin-Ring Fluorescent microspheres kit (1 *μ*m, F14791, Thermo Fisher). A fluorescence microscope (DMIL LED, Leica) was used for observation.

### 2.8. Western Blot Analysis

Protein was extracted and quantified using a BCA protein assay kit (Beyotime, China). Total protein was separated using 12% sodium dodecyl sulfate-polyacrylamide gel electrophoresis and transferred to polyvinylidene fluoride membranes. The membranes were blocked with a buffer containing 5% nonfat milk in PBS with 0.05% Tween-20 for 2 h and incubated with the primary antibody: anti-STAT3 antibody (1 : 1000, PAB30641, Bioswamp), anti-p-STAT3 (1 : 2000, ab76315, Abcam), anti-JAK (1 : 2000, PAB30711, Bioswamp), anti-p-JAK (1 : 2000, ab108596, Abcam), and anti-GAPDH (1 : 1000, PAB36269, Bioswamp) antibody. After three washes with PBS/Tween-20, the membranes were incubated with horseradish peroxidase-conjugated secondary goat antirabbit IgG (1 : 20000, SAB43714, Bioswamp) for 2 h at 25°C. Protein bands were visualized by enhanced chemiluminescence color detection (Tanon-5200, TANON, China) and analyzed using the TANON GIS software.

### 2.9. Data Analysis and Statistics

All data are presented as the mean ± standard deviation. Statistical analyses were performed using SPSS 19.0, and GraphPad prism 5.0 was used to produce figures. Data were evaluated for statistical significance using one-way ANOVA. Statistical significance was set at *P* < 0.05.

## 3. Results

### 3.1. NAR Inhibited BV-2 Cell Proliferation

To determine the effect of NAR treatment on cell proliferation, we compared the OD values of samples from the control, model, and various NAR treatment groups after culturing for 4 h (Figure 1(a)). Compared to the control group, the viability of BV-2 cells was significantly increased after treatment with LPS (Figure 1(b)). Compared to the model group, the viability of BV-2 cells was significantly decreased after treatment with different doses of NAR (*P* < 0.05) (Figure 1(c)), suggesting that NAR inhibits BV-2 cell proliferation.

### 3.2. NAR Inhibits Inflammation in BV-2 Cells

ELISA was used to detect the effect of NAR on the inflammatory response of BV-2 cells. The results showed that, compared with the control group, IL-10 and IGF-1 were significantly decreased in the model group (*P* < 0.05), whereas the expression levels of IL-1*β*, IL-6, and TNF-*α* were significantly increased (*P* < 0.05) (Figure 2). Compared with the model group, expression levels of IL-10 and IGF-1 in the NAR (5, 10, and 20 *μ*M) groups were significantly increased (*P* < 0.05), while those of IL-1*β*, IL-6, and TNF-*α* were significantly decreased (*P* < 0.05) (Figure 2). To examine the effect of NAR treatment on BV-2 cell activation, we performed assays to detect the microglial M1 and M2 phenotype markers iNOS and arginase 1, respectively [7]. Compared with the control group, the expression of iNOS increased in the model group but decreased following NAR treatment (Figure 3). Conversely, the level of arginase 1 increased after treatment with different doses of NAR (Figure 4), suggesting that NAR can promote the activation of BV-2 microglia towards the M2 phenotype.

### 3.3. NAR Inhibits BV-2 Cell Migration and Promotes BV-2 Cell Phagocytosis

We used a scratch test to observe the effect of NAR treatment on the migration of BV-2 cells. At 0 h postscratch, cells in all groups were similarly distributed, with minimal cells present in the scratched area (Figure 5(a)). By 24 h postscratch, we observed a nearly uniform distribution of cells in the model group in the scratched area, indicating cell migration (Figure 5(b)). Scratched area coverage was higher in the model group compared to the control group at this time. We observed that NAR treatment impaired migration compared to the model group, especially in the 10 *μ*M and 20 *μ*M treatment groups. A FocalCheck™ Thin-Ring Fluorescent Microspheres Kit was used to observe BV-2 cell phagocytosis. The phagocytic capacity of BV-2 cells was impaired after LPS treatment in the model group, whereas this impairment was alleviated following treatment with various concentrations of the NAR intervention, as demonstrated by the improved phagocytic capacity of NAR-treated BV-2 cells (Figure 6).

### 3.4. NAR Exerts its Protective Effects through the JAK/STAT3 Pathway

To study whether NAR functions through the JAK/STAT3 pathway, we used a JAK2 inhibitor (WP1066, 5 *μ*M) to perturb signaling and observed changes in the activation of M1 and M2 markers in BV-2 cells as well as JAK/STAT3 pathway-related factors. Compared with the control group, the expression of iNOS was increased in the model group (Figure 7). Compared with the model group, the expression of iNOS was decreased following NAR, NAR + WP1066, or WP1066 treatments (Figure 7), whereas the level of arginase 1 was increased (Figure 8). These changes were most pronounced in the NAR + WP1066 treatment group. Next, we detected the expression of p-STAT3 and p-JAK using Western blotting (Figure 9). Compared with the control group, the protein expression levels of p-STAT3 and p-JAK in the model group were significantly increased (*P* < 0.05). Compared with the model group, the protein expression levels of p-STAT3 and p-JAK in the NAR, NAR + WP1066, and WP1066 treatment groups were significantly decreased (*P* < 0.05), and the combined treatment of NAR + WP1066 resulted in a significant decrease in expression compared to NAR treatment alone (*P* < 0.05). These data suggest that NAR plays a protective role in BV-2 cells by inhibiting the JAK/STAT3 pathway.

## 4. Discussion

The immune system plays an important role in the relationships between sleep, health, and neurodevelopment [24, 25]. Clinical data show that sleep disorders, including insomnia, can cause immune dysfunction [1–4]. Sleep deprivation may increase the risk of inflammation and infection by altering immune function, whereas napping or extending sleep can restore immune system homeostasis [26, 27]. Various studies have reported that microglia became activated in the brains of sleep-deprived mice, and the number and morphology of microglia were significantly positively correlated with neuronal apoptosis [28, 29]. In this study, we found that NAR could effectively alleviate cell proliferation induced by LPS, suggesting that NAR may play a protective role by inhibiting microglia proliferation.

Activated microglia secrete TNF-*α*, IL-1*α*, and C1q to induce the differentiation of astrocytes towards the M1 phenotype. M1 astrocytes lose their ability to promote neuronal survival, growth, and synaptic formation and cause neuronal and oligodendrocyte cell death [13]. Following LPS treatment, we observed that the expression of the M1 marker iNOS and the cytokines IL-1*β*, IL-6, and TNF-*α* increased, while the expression of M2 marker arginase 1 was largely unchanged and the expression of IL-10 and IGF-1 decreased; these findings were consistent with previous reports [30]. However, following NAR treatment, the above results were reversed. The expression of iNOS, IL-1*β*, IL-6, and TNF-*α* decreased, while the expression of arginase 1, IL-10, and IGF-1 increased. This suggests that NAR treatment may preferentially promote the differentiation of microglia towards the M2 rather than the M1 phenotype. Additionally, we observed that NAR treatment significantly reversed the LPS-induced decrease in phagocytic function. Taken together, these data support the hypothesis that NAR can exert its protective effect by inhibiting cellular inflammation, promoting the differentiation of microglia to the M2 phenotype, and increasing phagocytosis.

Many signaling pathways are known to be involved in the activation of microglia, including MAPKs (ERK/P38/JNK), NF-*κ*B, JAK/STAT, and PI3K [31]. JAK/STAT3 has been reported to be activated in patients with sleep deprivation [32]. The JAK/STAT pathway in microglia is regulated by cytokines, such as IL-6, in the microenvironment and is directly involved in regulating the activity of neighboring cells (mainly astrocytes and neurons) [14–18]. We observed that inhibiting JAK/STAT signaling promoted the activation of microglia to M2 microglia.

In conclusion, NAR can inhibit the proliferation, migration, and inflammation of BV-2 cells; inhibit the activation of microglia to the M1 type; promote the activation of microglia to the M2 type; and enhance the phagocytic function of BV-2 cells. The effect may have been achieved by regulating the activity of the JAK/STAT3 pathway.

## Figures and Tables

**Figure 1:** Cell viability was detected using CCK8. (a) OD value for the different treatment groups. (b) Cell viability in the control and model groups, ^*∗*^*P* < 0.05 vs. Control. (c) Cell viability after 24 h of NAR treatment (5, 10, or 20 *μ*M) intervention, ^*∗*^*P* < 0.05 vs. model. *N* = 3.

**Figure 2:** Expression levels of IL-1*β*, IL-6, TNF-*α*, IL-10, and IGF-1 were quantified using ELISA. ^*∗*^*P* < 0.05 vs. control; ^#^*P* < 0.05 vs. model. *N* = 3.

**Figure 3:** iNOS immunofluorescence (green) in BV-2 cells with or without NAR treatment. Scale bar, 100 *μ*m.

**Figure 4:** Arginase 1 immunofluorescence (green) in BV-2 cells with or without NAR treatment. Scale bar, 100 *μ*m.

**Figure 5:** Effect of NAR treatment on the BV-2 cell migration. Brightfield images of cells with or without NAR treatment 0 h postscratch test (a) and 24 h postscratch test. (b) Scale bar, 250 *μ*m.

**Figure 6:** Effect of NAR treatment on BV-2 cell phagocytosis. Cell phagocytosis was observed using the FocalCheck™ Thin-Ring Fluorescent Microspheres Kit. Scale bar, 50 *μ*m.

**Figure 7:** iNOS immunofluorescence in BV-2 cells with or without NAR and/or WP1066 treatment. Scale bar, 100 *μ*m.

**Figure 8:** Arginase 1 immunofluorescence in BV-2 cells with or without NAR and/or WP1066 treatment. Scale bar, 100 *μ*m.

**Figure 9:** Western blot of p-STAT3 and p-JAK. ^*∗*^*P* < 0.05 vs. Control; ^#^*P* < 0.05 vs. Model; &*P* < 0.05 vs. NAR. *N* = 3.

## Data Availability

The data used to support the findings of this study are available from the corresponding author upon request.
